The article "The Influence of Traditional Culture Integration into Chinese Language and Literature Teaching on the Improvement of Mental Health of College Students" was published in 2022. Journal: J Environ Public Health.

# The Influence of Traditional Culture Integration into Chinese Language and Literature Teaching on the Improvement of Mental Health of College Students

**DOI:** 10.1155/2022/9528503

**Published:** 2022-09-15

**Authors:** Yuanyuan Zheng

**Affiliations:** School of Languages and Media, Anhui University of Finance and Economics, Bengbu 233030, China

## Abstract

Contemporary college students not only face the pressure brought by their studies but also bear the pressure brought by society and their families. Helping college students correctly understand their mental health and effectively solve their' mental health diseases has become an important issue in education research. The cultivation of healthy psychological quality is inseparable from the cultivation of a humanistic spirit. Therefore, integrating excellent traditional culture into Chinese language and literature teaching and research and giving full play to and inheriting the educational role of excellent traditional culture can not only improve the literary quality of college students and benefit the construction of healthy mental of college students. The main purpose of this research is to analyze the effect of Chinese excellent traditional culture on the cultivation of college students' mental health, analyze the impact of traditional culture integration into Chinese language and literature teaching research on improving college students' mental health, and propose the valuable suggestion for integration of excellent traditional culture into Chinese language and literature teaching research. Firstly, we analyze the benefits of integrating traditional culture in literature to the construction of college students' healthy psychology; then, the current deficiencies of literature education are analyzed; next, through literature analysis and summary, the main factors affecting the mental health of college students were found and the importance of these factors was evaluated by questionnaire survey and mathematical statistics methods; finally, targeted opinions and suggestions are put forward. This research provides guidance and reference for inheriting excellent national culture through literature education and constructing university health psychology in the future.

## 1. Introduction

The rapid social and economic development and the gradual improvement of people's living standards have provided contemporary college students with a broad development platform and bright prospects but also brought them certain temptations and challenges [1, 2]. Contemporary college students are in an important period of growth, and their physiology and psychology are not yet fully mature [3, 4]. Although they are optimistic and cheerful, love life, and have a strong sense of responsibility to the society, psychological imbalance and moral anomie often appear in them [5]. It has become an urgent problem to be solved in the mental health education of college students [6, 7]. Although China's understanding of college students' mental health education has gradually deepened over the past ten years and the practice has been continuously strengthened, the current situation shows that mental health education has little effect. The future world belongs to young college students, and college students are responsible for national revitalization and national prosperity. In the construction of socialist modernization, while educating college students on patriotism and professional knowledge, inherit and carry forward the spirit of China's excellent traditional culture, learn from its moral education methods, has significant theoretical and practical significance for college students form socialist core values and life for college students under the conditions of a market economy [8, 9]. Only by identifying, affirming, and confident with the unique advantages, immortal charm, and values of our traditional culture can we be confident in the system, theory, and path of socialism with Chinese characteristics, and we can internalize the core socialist values in our hearts and actions [10]. Cultural self-confidence is the premise and support of institutional self-confidence, theoretical self-confidence, and road self-confidence [11, 12]. Under this background, colleges and universities, which shoulder the major task of cultivating morality and building talents, should vigorously carry forward Chinese traditional culture and fully tap the rich resources of traditional culture. The spirit of China's excellent traditional culture belongs to the positive and positive part of traditional culture and is the essence and core of traditional culture. Inheriting and developing Chinese traditional culture will surely inherit and develop the spirit of excellent traditional culture [13, 14].

The article "The Influence of Traditional Culture Integration into Chinese Language and Literature Teaching on the Improvement of Mental Health of College Students" was published in 2022. Journal: J Environ Public Health.

Although the mental health education of college students in our country develops rapidly and has many research achievements, in the process of its development, it is generally guided by mature western psychological theories [15, 16]. China is a big country of cultural development, and there are rich mental health education ideas in traditional culture, which have a good guiding role in the construction of positive and healthy college students' psychology. The construction of healthy psychology for local college students should be based on the fundamentals of China [17]. Although mature Western psychological theories have provided a favorable reference for my country's mental health education, there are still some shortcomings, which have led to the current lack of mental health education [18, 19]. The actual effect is not ideal, and it cannot really penetrate the hearts of students. In order to really improve the effectiveness of college students' mental health education and play its important role, it is very necessary to carry out innovative research on it and to apply the essence of traditional culture [20]. Only innovation can promote the better development of mental health education, and only based on traditional culture can it improve its pertinence and effectiveness [21]. During five thousand years of historical development, China has formed a broad and profound excellent culture, which contains rich philosophical thoughts, humanistic spirit, moral concepts, and value orientations. Buddhism, Taoism, and Confucianism, as the three main bodies of traditional culture, are widely accepted and inherited by people; they contain the main traditional thoughts and culture that have been circulated in China for 5000 years, covering a large number of historical and cultural common sense, historical allusions, and philosophical truths. Extracting and learning from the excellent ideas will not only help us enhance national cohesion and national pride but also help us cultivate our virtues and realization of the value of life. Confucianism advocates self-cultivation, family order, governance of the country, and peace in the world. Self-cultivation is the foundation of everything and advocates people to be proactive and make achievements [22]. Taoism advocates letting nature go with the flow, ruling by inaction, advocating safety and duty, indifference to fame and fortune, and attaching importance to the harmony between man and nature. Buddhists advocate loving all beings, selfless devotion, refraining from doing evil, practicing all kindness, abiding by the Ten Commandments, having peace of mind, and using wisdom [23]. Although their ideological emphases are different, their inner thoughts are the same, and they all take people as the starting point to realize the meaning of life [24]. And since the Tang Dynasty, there has been a theory of the unity of three religions, so this research will use the excellent qualities mentioned, such as loyalty, filial piety, courtesy, and honesty, in various traditional Chinese cultures as the representative of traditional culture for research.

A university is a place where ideas meet and where people are cultivated. Universities should also be a place for people to think about the meaning of human existence and the true meaning of learning, and the places and platforms that universities can provide for this should at least include literary education and research [25, 26]. At present, Chinese language and literature occupy an important position in our current various learning subjects, and it is also an important carrier of quality education at this stage [27]. By learning the Chinese language, one can deeply perceive the traditional culture of the Chinese nation and absorb a more profound national spirit [28, 29]. On the basis of the ideological value and humanistic feelings of our ancestors, actively absorbing advanced ideas has important guiding value for our study and life, helping us to improve our humanistic quality and enrich our spiritual world. The purpose of this study are (1) to analyze the mental health of college students, (2) to investigate the current situation and existing problems of the integration of traditional culture into Chinese language and literature teaching research, (3) to analyze its impact on improving the mental health of college students, and (4) to propose solutions to the existing problems. The research route is shown in Figure 1. First, review the literature and organize data to identify factors that may affect college students' mental health and analyze the current situation and shortcomings of moral education through literature synchronous; next, a questionnaire survey based on influencing factors obtained above is performed; finally, according to the result of this study, some effective recommendations are proposed.

The article "The Influence of Traditional Culture Integration into Chinese Language and Literature Teaching on the Improvement of Mental Health of College Students" was published in 2022. Journal: J Environ Public Health.

## 2. The Significance of Integrating Excellent Traditional Culture into Chinese Language and Literature Teaching on the Mental Health of College Students

### 2.1. Benefit for Improving Humanistic Quality

The content of the current Chinese language learning is rich, and different works contain the ancients' experience of nature and life and the pursuit of spiritual values. In-depth study of such traditional culture can not only improve the basic cultural quality of students but also allow us to deeply perceive more philosophy of life [30]. With the help of the ideological achievements of the ancients, we can face various confusions in current study and life and improve students' humanistic quality. Humanistic literacy is the basic quality, values, and code of conduct formed through learning and practical activities. At present, the content related to Chinese language and literature has penetrated various stages of quality education. The main purpose of learning Chinese language and literature is to master the foundation of Chinese language and literature and to improve reading comprehension, writing, and work appreciation. After accumulating to a certain extent, literary knowledge can be transformed into personal inner temperament, which can better show the charm of traditional Chinese literature; excellent quality in literary works can cultivate the sentiments of college students and cultivate their positive attitudes and play a critical role in the comprehensive development of college students in the future.

The article "The Influence of Traditional Culture Integration into Chinese Language and Literature Teaching on the Improvement of Mental Health of College Students" was published in 2022. Journal: J Environ Public Health.

### 2.2. Benefit for Improving the Quality of Thinking

Excellent language and literature work themselves have many excellent elements beyond the modern society, and they are also the epitome of our traditional culture [31]. Excellent culture can infect and guide our learners. Most of the important characters selected in the current Chinese language and literature works have noble characters. For example, when studying and appreciating the “Historical Records,” the personal biographies of many characters are recorded, and different events are of great educational value to us. Reading historical works related to “Shiji” can not only optimize the ideological and moral character of our learners but also help students establish lofty and lofty ideals in life, which is a concentrated expression of the important role of Chinese language and literature works. Through the influence of Chinese language and literature, our students can establish principles and moral standards in their learning, which plays an important role in guiding our college students' practical activities. With the example of learning, college students will be strict with themselves, and college students under the influence of excellent culture will have a positive mentality, thereby subtly cultivating a healthy attitude of college students.

### 2.3. Benefit for Enriching of Spiritual World

Chinese's traditional culture and national spirit are profound and longstanding and are also the main carrier of my country's academic education [32]. At present, the external environment we face in the education stage is relatively complex, and in the materialistic real society, students ignore the spiritual pursuit and only pursue the comfort of life. Through long-term Chinese language learning, we can seek the main direction of learning and pursue spiritual beliefs in the complex modern society. We will face many difficulties in our daily study and life. Through the extensive knowledge of traditional culture and Chinese language and literature works, we can provide more guidance for life, find ourselves in learning, reflect on ourselves, pursue the true meaning of life, and enrich our inner world and keep us from being corrupted by all kinds of bad ideas and values.

### 2.4. Benefit for Improving Humanistic Behavior

There are many excellent ideas in Chinese traditional culture, and these excellent ideas have influenced generations of Chinese people [33]. It is precisely because of the study of Chinese language, on the basis of following the social system of the rule of law, that the daily behavior of our students is regulated by advanced ideas and the all-around development of the society is promoted. After learning the value concept of “hundreds of kindness and filial piety first,” we can play a guiding role in various behaviors in life so that each of us can build sufficient ideological and moral power reserves in our hearts. Whether it is daily Chinese language learning or reading of excellent literary works, it is important in the establishment of advanced ideas and norms of behavior and can lay a good foundation for our comprehensive development in the future.

The article "The Influence of Traditional Culture Integration into Chinese Language and Literature Teaching on the Improvement of Mental Health of College Students" was published in 2022. Journal: J Environ Public Health.

## 3. The Problems and Research Methods in the Cultivation of Mental Health in the Literature Education and Research of Colleges

### 3.1. The Shortage in Existing Research

In recent years, the mental health of college students has received extensive attention from scholars, and more and more studies have combined it with traditional Chinese culture. After reviewing many research results, it is found that there are certain deficiencies.

Most of the research on positive psychological qualities in traditional culture is presented in the form of theory, and the research on this is still in the stage of speculative discussion, mostly the interpretation of classic works in traditional culture. These studies mainly use the methods of logical speculation, literature analysis, and experience summarization, their theories are not deep enough, and there are few creative literature [34, 35]. In addition, most of these literatures are qualitative descriptions, lacking quantitative analysis of the impact of various qualities on college students.

Most of the researchers on positive thoughts and positive psychological qualities in traditional culture belong to philosophy, sociology, or education, and relatively few studies have been done on them from the perspective of literature [36, 37]. Little research has been done in this area. Research on the effect of positive psychological quality on college students' positive psychology in traditional cultures is particularly rare. The research on positive psychological quality is mainly concentrated in the field of mental health, and most of them are from the perspectives of ideological and political education and philosophy. It is important for building socialist values. Implanting traditional excellent culture in literature education can subtly affect the personality of college students, which can be of great help to college students' mental health. Therefore, it is particularly necessary to analyze the influence of traditional culture integration into literature education research on the positive psychology of Chinese college students.

The article "The Influence of Traditional Culture Integration into Chinese Language and Literature Teaching on the Improvement of Mental Health of College Students" was published in 2022. Journal: J Environ Public Health.

### 3.2. The Research Methods of This Study

This research takes Chinese traditional culture as the main starting point, extracts the excellent qualities, and understands the influence of traditional culture integration into literature teaching research on the mental health of college students. First of all, we compiled a psychological quality evaluation scale, carried out item analysis, and used exploratory factor analysis to test and correct the dimensions of the prediction scale to form the final positive psychological quality scale. Then, the current situation of the positive psychological quality of college students is investigated, and the relationship between the integration of excellent traditional culture in literacy education and the psychological health of college students is analyzed.

The innovation of this research is illustrated in two aspects. In the first aspect, from the perspective of literary education research, we study the influence of excellent quality in traditional culture on college students' psychological well-being, not only limited to theoretical research but also trying to obtain new insights from research Second, for the combination of literature education research and traditional culture, it is mainly based on the positive factors in traditional culture, defines and studies the positive psychological quality from the original perspective of traditional culture, and provides a new perspective for the combination of them. In this study, quantitative analysis was used to obtain important procedures of factors affecting college students' mental health and then to cultivate college students' mental health by teaching students in accordance with their aptitude.

## 4. A Survey of College Students' Demand for the Excellent Quality of Traditional Culture

The purpose of this study is to explore the overall situation of the positive psychological quality of the selected sample college students through the questionnaire survey method and the self-compiled college students' positive psychological quality scale and to explore whether each dimension in the scale has obvious differences in various demographic variables, to provide data support for further research on the spiritual qualities required for cultivating college students' mental health in literary education. The impact factors to be investigated are determined through the literature survey method. According to the retrieval strategy, we searched the Web of Science for relevant literature, 901 articles were initially retrieved, and then 44 articles were finally included after heavy-duty and screening. A total of 179,469 college students were surveyed. The evaluation scores were 35 articles ranging from 4 to 7 points, and 3 articles were 8 points, which belonged to the medium- and high-quality literature.  Figure 2 shows the specific screening process.

The article "The Influence of Traditional Culture Integration into Chinese Language and Literature Teaching on the Improvement of Mental Health of College Students" was published in 2022. Journal: J Environ Public Health.

Before analyzing the data, it is necessary to divide the dataset and turn the disordered data into order. The change of information before and after dividing the dataset becomes the information gain, and then, the information gain obtained after each feature is divided into the dataset can be calculated, and it is the best choice to obtain the feature with the highest information gain.

Information entropy:

(1) $$\begin{array}{c} \text{Info}\left(D\right)=-\overset{m}{\underset{i=1}{\sum }}p_{i}\log_{2}\left(p_{i}\right). \end{array}$$

Information entropy after feature division:

(2) $$\begin{array}{c} {\text{Info}}_{R}\left(D\right)=\overset{k}{\underset{j=1}{\sum }}p_{i}\frac{\left|D_{j}\right|}{\left|D\right|}\times \text{Info}\left(D_{j}\right). \end{array}$$

Information gain:

(3) $$\begin{array}{c} \text{Gain}\left(R\right)=\text{Info}\left(D\right)-{\text{Info}}_{R}\left(D\right). \end{array}$$

To analyze the data in the literature, the random forest algorithm was used to analyze the factors that need to be investigated in this study; the algorithm flowchart is shown in Figure 3; and gender, specialization, grade, birthplace, and whether an only child are the variables of this study. The random forest algorithm has various implementation methods such as bootstrap sampling and bagging. In a process of bootstrap sampling, suppose there is currently a dataset *D* with *m* samples, and we perform *m* random sampling with “replacement” on it; in each round of sampling, the probability of sample *x* being drawn is 1/*m*, so after *m* rounds of sampling, the probability that the sample has not been drawn is

(4) $$\begin{array}{c} \underset{m⟶\infty }{\lim}{\left(1-\frac{1}{m}\right)}^{m}\approx \frac{1}{e}\approx 0.368. \end{array}$$

That is to say, about 36.8% of the samples in the original dataset were not drawn. When the data is large, the bagging method should be used. This method includes three steps.

The first step, input training times, the training set

(5) $$\begin{array}{c} D=\left\{\left(x_{1},y_{1}\right),\left(x_{2},y_{2}\right),\cdots ,\left(x_{m},y_{m}\right)\right\}. \end{array}$$

Training algorithm

(6) $$\begin{array}{c} h=I\left(D,D_{bs}\right). \end{array}$$

The second step, data processing, process is realized by a loop program, which is written as

(7) $$\begin{array}{c} \text{for }t=1,2,3,\cdots ,T,\\ h\left(t\right)=I\left(D,D_{bs}\right), \end{array}$$

end.

The article "The Influence of Traditional Culture Integration into Chinese Language and Literature Teaching on the Improvement of Mental Health of College Students" was published in 2022. Journal: J Environ Public Health.

Finally, the output is

(8) $$\begin{array}{c} H\left(x\right)=\arg\underset{y\in Y}{\max}\prod \left(h_{t}\left(x\right)=y\right). \end{array}$$

Unlike standard AdaBoost, which can only be used for binary classification tasks, bagging can be used for multiclassification, regression, and other tasks without modification.

To grasp the factors that affect students' personalities, it is also necessary to know which personality characteristics are most important to college students. AHP can solve this problem very well, and we found filial piety, kindness, courage, justice, fairness, probity, and creativity are the most important qualities college students need.

### 4.1. The Survey of College Students' Mental Health

College students from different regions were taken as subjects by means of a free online questionnaire. In total, 3000 questionnaires were distributed and 2570 valid questionnaires were recovered. They come from different institutions, including nationally renowned universities, local comprehensive institutions, and professional institutions. The detailed data information is shown in Table 1.

The subjects were tested by a self-made positive psychological quality scale, which consists of seven dimensions of filial piety, kindness, justice, integrity, fairness, courage, and creativity, with a total of 40 items. The scores of the questionnaires are assessed using Likert's five-point method, and the higher the score, the more positive psychological qualities it has. SPSS 24.0 was used to organize and analyze the obtained data. The total score obtained by the subjects on the positive psychological quality scale and the mean and standard deviation of the scores on each factor were counted, and the results are listed in Table 2. In addition, in order to show the difference in the scores of each factor more directly, the mean value of each factor is shown by a histogram in Figure 4. The total score of the positive psychological quality scale ranges from 24 to 120 points. In Table 2 and Figure 4, it is shown that the total score of the positive psychological quality of college students is 78.811, which is higher than the average level of theoretical scores. The positive psychological quality of the subjects was in the middle and upper level and had high positive psychological quality. Arranging the factors in descending order of average value, the order is filial piety, kindness, courage, justice, fairness, probity, and creativity. This shows that college students put filial piety in the first place in life and at the same time have kindness and care for others. Creativity ranks last, but its average value is not much different from probity and fairness, indicating that these three factors are less recognized than other factors.

The article "The Influence of Traditional Culture Integration into Chinese Language and Literature Teaching on the Improvement of Mental Health of College Students" was published in 2022. Journal: J Environ Public Health.

### 4.2. Difference Analysis of Demographic Variables of College Students' Positive Psychological Quality

The weight analysis of a single factor can provide teaching according to the different characteristics of college students, make up for the shortcomings of their mental health, and build a healthy psychology of college students in the fastest way. Analytic Hierarchy Process (AHP), a hierarchical weighted decision analysis method, is applied to analyze the significance of the demographic variables of college students. AHP is used to decompose the decision-making problem into different hierarchical structures in the order of the overall objective, subobjectives, evaluation criteria, and specific investment plans and then use the method of solving the eigenvectors of the judgment matrix to obtain the priority weight of an element to an element at the previous level, and the final weighted sum method is to recursively merge the final weight of each alternative to the total goal, and the one with the largest final weight is the optimal plan.

The judgment matrix has the following properties:

(9) $$\begin{array}{c} a\left(i,j\right)=\frac{1}{a\left(j,i\right)}, \end{array}$$

where *a*(*i*, *j*) is the comparison result of the importance of element *i* and element *j*, and the matrix formed by the pairwise comparison results is called the judgment matrix. The consistency index is calculated by CI.

(10) $$\begin{array}{c} \text{CI}=\frac{\lambda_{\max}\left(A\right)-n}{n-1}, \end{array}$$

where *n* is the order of the matrix and *λ* is eigenvalues, calculated by

(11) $$\begin{array}{c} \lambda_{\max}=\overset{n}{\underset{i=1}{\sum }}\frac{\lambda_{i}}{n}, \end{array}$$

(12) $$\begin{array}{c} \lambda_{i}=\overset{n}{\underset{i=j}{\sum }}\frac{a_{ij}w_{j}}{w_{i}}. \end{array}$$

The random consistency index RI is proposed to evaluate CI:

(13) $$\begin{array}{c} \text{RI}=\frac{{\text{CI}}_{1}+{\text{CI}}_{1}+\cdots +{\text{CI}}_{n}}{n}. \end{array}$$

Considering that the deviation of consistency may be caused by random reasons, a test coefficient CR is necessary:

(14) $$\begin{array}{c} \text{CR}=\frac{\text{CI}}{\text{RI}}. \end{array}$$

Generally, if CR < 0.1, it means the result is consistent; otherwise, it means the result is not satisfactorily consistent.

#### 4.2.1. Gender Difference Analysis

Taking gender as an independent variable, the total score of the positive psychological quality scale, and the scores on each factor as the dependent variable, the results of data analyses are shown in Figure 5 and listed in Table 3. It can be concluded from the table that there is no significant gender difference in the overall, but the total score of positive psychological quality of girls is slightly higher than that of boys. There are significant gender differences in the dimensions of benevolence and justice. Girls score higher on the benevolence dimension than boys, indicating that girls are more fraternal and compassionate than boys, while boys score higher than girls on the justice dimension, indicating that boys handle things more rational, more reemphasize loyalty.

The article "The Influence of Traditional Culture Integration into Chinese Language and Literature Teaching on the Improvement of Mental Health of College Students" was published in 2022. Journal: J Environ Public Health.

#### 4.2.2. Major Difference Analysis

The result of major difference analysis is shown in Figure 6 and listed in Table 4. The results of the study show that there is only a significant difference in the dimension of filial piety between science and engineering and literature and history college students, and there is just a small difference in different majors of the total score and the score of other factors. Students of literature and history are more filial than students of science and engineering.

#### 4.2.3. Grade Difference Analysis

The results of grade difference analysis are shown in Figure 7 and listed in Table 5. It can be seen from the table that there is no significant difference in the total score of the positive psychological quality of college students of different grades, but there are significant differences in the two dimensions of fairness and courage.

#### 4.2.4. Birthplace Difference Analysis

Taking the place of birth as an independent variable, the total score of the positive psychological quality scale and the score on each factor are used as the dependent variable to conduct an independent sample test.  Figure 8 and Table 6 show the results of this analysis. From Table 6, it can be concluded that there is no significant difference in the total score between rural and urban college students. However, there are significant differences in the dimensions of filial piety and courage. On the dimension of filial piety, college students from rural areas score higher, and college students from urban areas have more courage.

#### 4.2.5. Analysis of the Impact of Whether an Only Child

Whether the child is the only child of a family is taken as an independent variable for the difference analysis, and the conclusion is shown in Figure 9 and listed in Table 7. Overall, there is no significant difference between only child and non-only child, but there are significant differences in the dimensions of fairness, kindness, and integrity. College students who are not an only child have higher average scores in the dimensions of kindness and integrity, indicating that they are more helpful to each other, have a spirit of solidarity and love, and are more committed to their commitments. The average score of the only child is better in the dimension of fairness, indicating that they pay more attention to the distribution of resources and the maintenance of their own power.

The article "The Influence of Traditional Culture Integration into Chinese Language and Literature Teaching on the Improvement of Mental Health of College Students" was published in 2022. Journal: J Environ Public Health.

### 4.3. Analysis of the Results of the Survey

The total score obtained by the subjects on the positive psychological quality scale and the mean and standard deviation of the scores on each factor were counted, and the results are shown in Table 2. The total score of the positive psychological quality scale ranges from 24 to 120 points. Table 2 shows that the average total score of the positive psychological quality of college students is 78.811, which is higher than the average level of theoretical scores. The positive psychological quality of the subjects was in the middle and upper level and had a high positive psychological quality. Further analyze the factors in the positive psychological quality table, and arrange them in order of magnitude according to the average score of each factor. Filial piety is in the first place. Filial piety is a unique culture of our country. We were taught from childhood that “filial piety comes first,” which is also an important criterion for us to measure a person. The second is the dimension of benevolence. “Benevolence” is the main core of Confucius' thought, which brought changes to the society at that time. In today's society, the cultivation of one's own ideological and moral character and the harmonious coexistence of people and people and society also have guiding significance. The top two rankings in these two dimensions indicate that contemporary college students are still deeply influenced by traditional Chinese culture. Culture has long-term inheritance, and the influence of traditional Chinese culture on Chinese people has always existed. The second is courage. In today's increasingly convenient communication, we are exposed to more and more things, and traditional culture has gradually penetrated our lives. The rapid development of today's society has put forward higher requirements for us. Courage, enthusiasm, and curiosity have become increasingly important qualities. As for justice, a very important quality in traditional culture, sacrificing one's life for righteousness, courage to see righteousness, etc., it has been deeply rooted in the hearts of the people. Fairness, probity, and creativity rank in the bottom three of the seven dimensions, and the averages of the three dimensions are not much different. It is not that these dimensions are unimportant, but that in a society full of temptations, people pay too much attention to the result and ignore them in order to pursue the goals they want to achieve.

The article "The Influence of Traditional Culture Integration into Chinese Language and Literature Teaching on the Improvement of Mental Health of College Students" was published in 2022. Journal: J Environ Public Health.

## 5. The Influence of Integrating Traditional Culture into Literature Education and Research on the Construction of College Students' Psychology

These excellent spiritual qualities above-mentioned that college students' being need can be reflected in traditional Chinese culture. Therefore, it is feasible and necessary to use traditional culture in literature education to build healthy college students' psychology. There is a consensus on the concept of “literature as humanities.” Excellent literary works have a deep concern for people's living conditions and life values. Literary classics have a profound insight into the world we live in, penetrate the texture of human nature, illuminate the landscape of life, connect history, reality, and the future, and strike the hearts of generations of readers with beautiful expressions, profound thoughts, and broad minds. The resounding echoes span time and space and reach eternity. The fundamental purpose of literary education is to cultivate morality and cultivate people, and it focuses on the cultivation of personality and the cultivation of nonintelligence factors. It contains thinking about life and value orientation. To carry out literature education for students, we must stand on the standpoint of people, get rid of utilitarian thinking, and cultivate their aesthetic taste and aesthetic evaluation ability; to enrich students' spiritual world, pursuing the freshness of the soul and the richness of emotions; in imagination and experience based on cultivating the spirit of innovation, improve students' humanistic quality and aesthetic style. The influence of excellent culture can help college students form noble moral sentiments, maintain a positive attitude, and form a healthy psychology.

However, the teaching arrangement of basic education is aimed at examinations, and university education focuses on credits and employment. The purpose of students' studies seems to be to get into college with high marks and find a decent, high-paying job. To a certain extent, this ignores the development of education in the true sense and is too practical to deal with the rhythm of social change. Einstein said: “It is not enough to educate a person with professional knowledge. Through professional education, he can become a useful machine, but he cannot become a person who develops harmoniously.” Literary education plays a role in coordination and balanced effect. But in actual teaching, literature education is often regarded as a matter of the Chinese classroom. And Chinese classrooms often turn literature education into simple and rigid knowledge teaching. Practical language trainings such as characters, words, sentences, blunt value standards, and boring preaching make works with profound emotions, profound meanings, and vivid images lacking flesh and blood, and the ideals of life, aesthetic awareness, and individual imagination inherent in literature are all banished. At the university, literature education is considered to be only a matter of the Chinese Department and the Faculty of Letters. Students of other majors tend to keep an aloof and indifferent attitude toward literature. The lack of humanistic literacy represented by literary literacy affects the exploration of people's creative potential, and it is difficult to awaken the sense of life and value from the dormant self-consciousness and heart.

The article "The Influence of Traditional Culture Integration into Chinese Language and Literature Teaching on the Improvement of Mental Health of College Students" was published in 2022. Journal: J Environ Public Health.

Literature courses are set as public elective courses by colleges and universities because they are useless for employment, or they are generally canceled. Educators should let students understand that literary reading requires awareness of concepts and actions and that literary reading is related to life experience and spiritual enjoyment. It is necessary for students to fully feel and appreciate the joy brought by free and independent literary reading and pay attention to the value orientation and emotional standpoint of literary works. The student stage is the beginning of life and the budding stage of individual life. It needs the supply of knowledge to contribute to the society. Therefore, the humanistic spirit is needed to cultivate students' humanistic heritage and to shape good humanistic conduct, healthy mind, and correct personality. Literary education is a process of indoctrination, and in the process of educating people, it gives full play to the two functions of moral education and aesthetic education. Humanistic quality and moral education are different from each other, and they are related to each other and influence each other. Both belong to the category of literary education. Moral education is the direction mark of humanistic quality. In the process of literary education, the principle of moral education is abided by, the moral education factors of literary works are fully explored, and the cultivation of humanistic quality and moral education is carried out at the same time. Incorporating excellent traditional culture into literature education and teaching is an important way to cultivate students' humanistic quality, and it should be permeated in the teaching of various subjects, which can promote the improvement of students' abilities and the sublimation of emotions. According to the characteristics of different students, teach students in accordance with their aptitude, considering the students' major, gender, grade, whether they are an only child, and other factors, analyze their psychological characteristics, carry out mental health education in a targeted manner, build the healthy psychology of college students, and cultivate them into outstanding talents.

The article "The Influence of Traditional Culture Integration into Chinese Language and Literature Teaching on the Improvement of Mental Health of College Students" was published in 2022. Journal: J Environ Public Health.

## 6. Conclusions and Discussion

This study is based on the influence of the integration of literature education research into Chinese excellent traditional culture on the mental health of contemporary college students. Through the investigation of the existing literature and statistical analysis of their data, we found that seven factors, including filial piety, fairness, justice, kindness, courtesy, probity, and creativity, can be used as the main indicators to quantify the mental health of college students. Further, the above factors were evaluated based on differences in gender, major, grade, place of birth, and whether they were an only child by questionnaire survey and analysis of the data obtained by questionnaire survey through AHP. The results show that the mental health of college students is healthy overall, but there are differences in the scores of various factors, gender, grade, etc. In addition, the insufficiency of integrating traditional culture in literary education is analyzed and found that current literature education pays too much attention to knowledge and neglects moral education. Integrating traditional culture into literature education can cultivate the positive and healthy psychology of college students, which also can subtly affect the daily behavior of students, and it will inevitably change the mental health of students from external performance to inner self-restraint, thereby building a healthy college student psychology. Combined with the previous research results of experts and scholars, this paper discusses the current situation of college students' positive psychological quality and the relationship between college students' psychological health and literature education and puts forward a new way for constructing positive psychological quality of college students, students should be taught by their aptitude, and ideological education should be carried out according to the gender, origin, grade, etc. of the student group, to help them become talents. This study tries to create a new perspective on positive psychological quality research and at the same time provides a reference for literature teaching research. Traditional culture is extensive and profound. This research only initially explores several representative dimensions and selects several topics as representatives for measurement. There are great limitations. We should deepen the understanding of traditional culture, create more dimensions, and construct more rigorous topics and detailed and in-depth research. The discussion on the integration of traditional culture into literature is also not deep enough, and more in-depth research will be done in these areas in the future.

The article "The Influence of Traditional Culture Integration into Chinese Language and Literature Teaching on the Improvement of Mental Health of College Students" was published in 2022. Journal: J Environ Public Health.

## Figures and Tables

**Figure 1:** Technology roadmap.

**Figure 2:** Literature screening process.

**Figure 3:** Schematic diagram of random forest algorithm.

**Figure 4:** Scores for main factors that affect college students' mental health.

**Figure 5:** Scores for college students of different gender.

**Figure 6:** Scores for college students of different major.

**Figure 7:** Scores for college students of different grade.

**Figure 8:** Scores for college students of different birthplace.

**Figure 9:** Scores for college students whether an only child.

**Table 1:** Information distribution table of demographic variables.

	Variables	Number	Percentage
Gender	Male	1195	46.5
	Female	1375	53.5

Specialized	Science and engineering	1050	40.9
	Literature and history	1520	59.1

Grade	Freshman	650	25.3
	Sophomore	640	24.9
	Junior year	650	25.3
	Senior year	630	24.5

Birthplace	City	1580	61.5
	Countryside	990	38.5

Only child	Yes	1165	45.3
	No	1405	54.7

**Table 2:** Total score and the mean and standard deviation of each factor (*n* = 2570).

	Mean value	Standard deviation
Filial piety	4.339	0.5329
Kindness	3.721	0.6383
Courage	3.528	0.8054
Justice	3.040	0.7738
Fairness	2.703	0.7590
Probity	2.695	0.6392
Creativity	2.626	0.8782
Total score	78.811	7.6531

**Table 3:** Gender difference analysis.

	Male	Female	*t*	*p*
Filial piety	4.312 ± 0.6238	4.364 ± 0.5734	-0.694	0.256
Fairness	2.694 ± 0.6839	2.706 ± 0.6468	-0.274	0.449
Justice	3.093 ± 0.6914	2.924 ± 0.6217	3.887	0.002
Kindness	3.638 ± 0.7926	3.831 ± 0.6366	-4.295	0.001
Courage	3.638 ± 0.7926	3.532 ± 0.7478	-0.443	0.371
Probity	2.662 ± 0.7290	2.751 ± 0.6971	-1.628	0.055
Creativity	2.631 ± 0.6334	2.622 ± 0.6192	0.268	0.451
Total score	78.247 ± 9.4726	79.056 ± 7.9352	-1.623	0.067

**Table 4:** Major difference analysis.

	Literature and history	Science and engineering	*t*	*p*
Filial piety	4.402 ± 0.6228	4.264 ± 0.6182	2.753	0.031
Fairness	2.700 ± 0.7396	2.705 ± 0.6924	-0.046	0.971
Justice	3.033 ± 0.6297	3.052 ± 0.5903	-0.309	0.318
Kindness	3.747 ± 0.5893	3.683 ± 0.7430	0.775	0.178
Courage	3.547 ± 0.8241	3.513 ± 0.6475	0.461	0.391
Probity	2.701 ± 0.7392	2.697 ± 0.6391	0.659	0.443
Creativity	2.654 ± 0.6032	2.569 ± 0.6765	1.351	0.059
Total score	79.322 ± 8.9833	78.274 ± 9.6401	2.525	0.056

The article "The Influence of Traditional Culture Integration into Chinese Language and Literature Teaching on the Improvement of Mental Health of College Students" was published in 2022. Journal: J Environ Public Health.

**Table 5:** Grade difference analysis.

	Freshman	Sophomore	Junior year	Senior year	*F*	*p*
Filial piety	4.362 ± 0.645	4.331 ± 0.615	4.405 ± 0.509	4.336 ± 0.710	1.412	0.294
Fairness	2.621 ± 0.728	2.697 ± 0.674	2.710 ± 0.625	2.734 ± 0.743	7.865	0.000
Justice	3.147 ± 0.661	2.985 ± 0.728	3.048 ± 0.753	3.004 ± 0.621	1.095	0.325
Kindness	3.653 ± 0.589	3.741 ± 0.791	3.711 ± 0.649	3.692 ± 0.677	1.167	0.319
Courage	3.698 ± 0.723	3.732 ± 0.592	3.433 ± 0.663	3.448 ± 0.712	3.877	0.009
Probity	2.703 ± 0.813	2.690 ± 0.640	2.712 ± 0.728	2.691 ± 0.636	0.932	0.430
Creativity	2.634 ± 0.717	2.613 ± 0.711	2.601 ± 0.678	2.629 ± 0.667	0.189	0.923
Total score	78.321 ± 9.164	79.024 ± 11.23	78.907 ± 15.57	79.321 ± 12.87	0.986	0.553

**Table 6:** Birthplace difference analysis.

	City	Countryside	*t*	*p*
Filial piety	4.346 ± 0.5278	4.331 ± 0.6132	3.045	0.027
Fairness	2.702 ± 0.6309	2.709 ± 0.7291	-0.286	0.512
Justice	3.038 ± 0.6281	3.059 ± 0.6478	-0.458	0.461
Kindness	3.742 ± 0.7013	3.712 ± 0.6254	0.984	0.249
Courage	3.461 ± 0.6794	3.558 ± 0.7325	-1.443	0.045
Probity	2.706 ± 0.6537	2.691 ± 0.6172	0.266	0.469
Creativity	2.630 ± 0.6667	2.627 ± 0.7903	0.213	0.533
Total score	79.003 ± 9.3752	78.734 ± 10.3417	1.823	0.084

**Table 7:** Difference analysis of the dimension of only child.

	Yes	No	*t*	*p*
Filial piety	4.335 ± 0.6461	4.342 ± 0.5839	-1.332	0.063
Fairness	2.637 ± 0.7462	2.776 ± 0.6327	2.294	0.037
Justice	3.030 ± 0.7294	3.043 ± 0.6291	0.275	0.532
Kindness	3.556 ± 0.7434	3.743 ± 0.6865	-2.823	0.031
Courage	3.532 ± 0.6907	3.525 ± 0.6281	0.378	0.529
Probity	2.688 ± 0.8339	2.705 ± 0.7326	-1.734	0.046
Creativity	2.573 ± 0.7242	2.665 ± 0.9367	0.830	0.073
Total score	78.305 ± 13.7821	79.947 ± 9.4365	-1.232	0.104

## Data Availability

The datasets used during the current study are available from the corresponding author on reasonable request.

## References

[1] Wang Q. (2014). Effects of urbanisation on energy consumption in China. *Energy Policy*.

[2] Wang Y. S., Xie Z., Wu R., Feng K. (2022). How does urbanization affect the carbon intensity of human well-being? A global assessment. *Applied Energy*.

[3] Vereecke S., Sorensen K., Zhu J. (2022). The impact of physical conditions on the incidence of major depressive disorder in Chinese university students: results from a longitudinal study. *Journal of Affective Disorders*.

[4] Mao Y., Zhang N., Liu J., Zhu B., He R., Wang X. (2019). A systematic review of depression and anxiety in medical students in China. *BMC Medical Education*.

[5] Fu W., Yan S., Zong Q. (2021). Mental health of college students during the COVID-19 epidemic in China. *Journal of Affective Disorders*.

The article "The Influence of Traditional Culture Integration into Chinese Language and Literature Teaching on the Improvement of Mental Health of College Students" was published in 2022. Journal: J Environ Public Health.

[6] Zhang M. X., Mou N. L., Tong K. K., Wu A. M. S. (2018). Investigation of the effects of purpose in life, grit, gratitude, and school belonging on mental distress among Chinese emerging adults. *International Journal of Environmental Research and Public Health*.

[7] Zou P., Sun L., Yang W. (2018). Associations between negative life events and anxiety, depressive, and stress symptoms: a cross-sectional study among Chinese male senior college students. *Psychiatry Research*.

[8] Jung J. (2018). Young women’s perceptions of traditional and contemporary female beauty ideals in China. *Family and Consumer Sciences Research Journal*.

[9] Xu Z., Zou D., Wu C.-H. (2022). Big data analysis research on the deep integration of intangible cultural heritage inheritance and art design education in colleges and universities. *Mobile Information Systems*.

[10] Chan R. C. H. (2022). A social cognitive perspective on gender disparities in self-efficacy, interest, and aspirations in science, technology, engineering, and mathematics (STEM): the influence of cultural and gender norms. *International Journal of STEM Education*.

[11] Priestley M., Hall A., Wilbraham S. J., Mistry V., Hughes G., Spanner L. (2022). Student perceptions and proposals for promoting wellbeing through social relationships at university. *Journal of Further and Higher Education*.

[12] Pedler M. L., Willis R., Nieuwoudt J. E. (2021). A sense of belonging at university: student retention, motivation and enjoyment. *Journal of Further and Higher Education*.

[13] Weng L., Zhang Y. B., Kulich S. J., Zuo C. (2021). Cultural values in Chinese proverbs reported by Chinese college students. *Asian Journal of Social Psychology*.

[14] Hu X., Chen S. X., Zhang L., Yu F., Peng K., Liu L. (2018). Do Chinese traditional and modern cultures affect young adults’ moral priorities?. *Frontiers in Psychology*.

[15] Tay A. K., Riley A., Islam R. (2019). The culture, mental health and psychosocial wellbeing of Rohingya refugees: a systematic review. *Epidemiology and Psychiatric Sciences*.

[16] Kpanake L. (2018). Cultural concepts of the person and mental health in Africa. *Transcultural Psychiatry*.

[17] Copeland W. E., McGinnis E., Bai Y. (2021). Impact of COVID-19 pandemic on college student mental health and wellness. *Journal of the American Academy of Child & Adolescent Psychiatry*.

[18] Auerbach R. P., Mortier P., Bruffaerts R. (2019). Mental disorder comorbidity and suicidal thoughts and behaviors in the World Health Organization world mental health surveys international college student initiative. *International Journal of Methods in Psychiatric Research*.

[19] Karyotaki E., Cuijpers P., Albor Y. (2020). Sources of stress and their associations with mental disorders among college students: results of the World Health Organization world mental health surveys international college student initiative. *Frontiers in Psychology*.

The article "The Influence of Traditional Culture Integration into Chinese Language and Literature Teaching on the Improvement of Mental Health of College Students" was published in 2022. Journal: J Environ Public Health.

[20] Lattie E. G., Lipson S. K., Eisenberg D. (2019). Technology and college student mental health: challenges and opportunities. *Frontiers in Psychiatry*.

[21] Kalkbrenner M. T., Jolley A. L., Hays D. G. (2019). Faculty views on college student mental health: implications for retention and student success. *Journal of College Student Retention: Research, Theory & Practice*.

[22] Yongli L., Yiping L. (2021). Self-cultivation as the basis of person making: a Confucian perspective illustrated by a case study of Zeng Guofan. *Psychology and Developing Societies*.

[23] Peters M. A. (2020). Educational philosophies of self-cultivation: Chinese humanism. *Educational Philosophy and Theory*.

[24] Buskell A. (2020). Cumulative culture and complex cultural traditions. *Mind & Language*.

[25] Roberts T., Jackson C., Mohr-Schroeder M. J. (2018). Students’ perceptions of STEM learning after participating in a summer informal learning experience. *International Journal of STEM Education*.

[26] McLure F. I., Fraser B. J., Koul R. B. (2022). Structural relationships between classroom emotional climate, teacher–student interpersonal relationships and students’ attitudes to STEM. *Social Psychology of Education*.

[27] Hansen M. H., Li H., Svarverud R. (2018). Ecological civilization: interpreting the Chinese past, projecting the global future. *Global Environmental Change*.

[28] Kwan L. Y. Y., Leung A. K. Y., Liou S. (2018). Culture, creativity, and innovation. *Journal of Cross-Cultural Psychology*.

[29] Mayer M. (2018). China’s historical statecraft and the return of history. *International Affairs*.

[30] Cindori S., Tolstova O., Levasheva Y. (2019). Humanistic trend in education in a global context. *SHS Web of Conferences*.

[31] Kim S., Raza M., Seidman E. (2019). Improving 21st-century teaching skills: the key to effective 21st-century learners. *Research in Comparative and International Education*.

[32] Ahmed A., Arshad M. A., Mahmood A., Akhtar S. (2019). The influence of spiritual values on employee’s helping behavior: the moderating role of Islamic work ethic. *Journal of Management, Spirituality & Religion*.

[33] Bedford O., Yeh K. H. (2019). The history and the future of the psychology of filial piety: Chinese norms to contextualized personality construct. *Frontiers in Psychology*.

[34] Carroll C., Hurry J. (2018). Supporting pupils in school with social, emotional and mental health needs: a scoping review of the literature. *Emotional and Behavioural Difficulties*.

The article "The Influence of Traditional Culture Integration into Chinese Language and Literature Teaching on the Improvement of Mental Health of College Students" was published in 2022. Journal: J Environ Public Health.

[35] McCloud T., Bann D. (2019). Financial stress and mental health among higher education students in the UK up to 2018: rapid review of evidence. *Journal of Epidemiology and Community Health*.

[36] Kourgiantakis T., Sewell K., McNeil S. (2019). Social work education and training in mental health, addictions and suicide: a scoping review protocol. *BMJ Open*.

[37] Mackie S. A., Bates G. W. (2018). Contribution of the doctoral education environment to PhD candidates’ mental health problems: a scoping review. *Higher Education Research & Development*.

